This article has been retracted.

# Clinical Potential of miR-451 and miR-506 as a Prognostic Biomarker in Patients with Breast Cancer

**DOI:** 10.1155/2022/9578788

**Published:** 2022-01-11

**Authors:** Yu Du, Zhuang Miao, Lijuan Qiu, Yan Lv, Kedi Wang, Lusheng Guo

**Affiliations:** ^1^Department of Laboratory, Beijing Friendship Hospital, Capital Medical University, Beijing City 100050, China; ^2^Department of Laboratory, Affiliated Hospital of Jilin Medical College, Jilin City 132013, Jilin Province, China; ^3^Department of Blood Transfusion, Beijing Children's Hospital, Capital Medical University, Beijing City 100045, China; ^4^Department of Laboratory, Beijing Public Security Hospital, Beijing City 100050, China

## Abstract

**Background:**

The incidence and mortality of breast cancer in the world remain high. The function and important role of miR-451 and miR-506 in a series of cancers have been proved. The purpose of this research was to explore the clinical diagnosis and prognostic significance of miR-451 and miR-506 expression in breast cancer.

**Methods:**

Quantitative real-time polymerase chain reaction (qRT-PCR) was applied to detect miR-451 and miR-506 expression in serum and tissues. The relationship of miR-451 and miR-506 with clinical parameters was determined by the chi-square test. Receiver operating characteristics (ROC) analysis was conducted to evaluate the diagnostic accuracy of miR-451 and miR-506 in breast cancer. In addition, we determined the prognostic performance of miR-451 and miR-506 using Kaplan–Meier survival assay.

**Results:**

The expression of miR-451 and miR-506 in breast cancer patients was significantly lower than that in healthy people. miR-451 and miR-506 expression decreased in breast cancer tissues compared with paracancerous tissue. High expression of miR-451 and miR-506 was associated with positive lymph node metastasis and late tumor node metastasis stage. Breast cancer patients with high miR-451 and miR-506 expression had lower five-year survival rate. The level of miR-451 and miR-506 expression showed high diagnostic accuracy for distinguishing breast cancer patients and healthy people.

**Conclusion:**

miR-451 and miR-506 could be used as biomarker for the diagnosis and prognosis of breast cancer.

## 1. Introduction

Breast cancer, one of the most frequent malignant tumors throughout the world, is the second and fifth most common cancer-induced female mortality in the USA and China, respectively [1, 2]. The incidence rate of breast cancer is currently the highest in the incidence rate of cancer. According to 2018 survey data from the International Agency for Research on Cancer (IARC), the incidence rate of breast cancer is 24.2% and 52.9% in developing countries [3, 4]. Despite the progress of early diagnosis, radiotherapy, and chemotherapy have been made, the high recurrence rate and low cure rate of advanced breast cancer are still a big problem [5]. Molecular biology has become the basis for developing personalized analysis for each patient. In recent years, more and more studies are focusing on identifying tumor biomarkers or therapeutic targets to enhance early diagnosis and treatment of breast cancer. Therefore, it is still very important to pay attention to identify novel factors for the prediction and effective treatment of breast cancer.

Since microRNA (miRNA) was first discovered in 1993, the miRNAs have gained more and more attention for their role in cell development and tumor [6]. miRNAs are single-stranded noncoding RNAs of 18–24 nucleotides in length and regulate protein synthesis in vivo by inhibiting the mRNA translation process by binding to the 3′-UTR region of the target gene [7]. Biological studies showed that miRNAs mainly affect the growth and progress of tumor cells through regulating the expression of target genes [8]. Studies have suggested a series of miRNAs abnormally expressed in breast cancer, such as miR-105-3p [9], miR-615-3p [10], and miR-485-5p [11], revealing they play a cardinal role in breast cancer. Moreover, the clinical significance of miRNAs in diagnosis and prognosis has also been proved in breast cancers, such as miR-940 [12], miR-4317 [13], and miR-1908-3p [14]. As the member of miRNAs, the vital role of miR-451 and miR-506 in some tumors has been proved [15, 16]. However, relationship between the expression of miR-451 and miR-506 and breast cancer diagnosis and prognosis has not yet been reported.

The purpose of the present study was to investigate the expression of miR-451 and miR-506 in serum and tissue, clarify the relationship between miR-451 and miR-506 and clinical features, and further measure their clinical value of diagnosis and prognosis in breast cancer patients.

## 2. Methods and Materials

### 2.1. Patients and Sample Collection

According to histopathological evaluation, 88 pairs of breast cancer tissue and corresponding adjacent nontumor tissue specimens were obtained from patients undergoing surgery from April to August 2018. Immediately after sampling, the tissue samples were put into liquid nitrogen and stored at −80°C for further experiments. Patients who underwent radiotherapy and chemotherapy before sampling were excluded. The clinical data of patients were obtained and recorded for further analysis, as given in Table 1. The staining results of estrogen receptor (ER) or progesterone receptor (PR) were considered to be positive when more than 10% cells were positive nuclear staining. The result for human epidermal growth factor receptor 2 (HER-2) staining was determined following the published UK guidelines [17]. The tumors were staged according to the 2009 Union for International Cancer Control (UICC) TNM system [18]. Sixty-three healthy volunteers without cancer were recruited from those who underwent routine physical examination. Venous blood samples were obtained from the patients and healthy controls in the same way in the morning after fasting for 8–10 h, and serum was obtained by centrifugation. All the serum samples collected were stored at −80°C for further analysis. The 5-year follow-up survival information was collected by telephone. The protocols were approved by the agency, and the consents to use their tissues for scientific research were all signed by patients.

### 2.2. RNA Extraction and Quantitative Real-Time Polymerase Chain Reaction (qRT-PCR)

MiRNeasy Serum/Plasma Kit (Qiagen, Germany) was applied to extract total serum RNA. After RNA concentration and purity determination (OD260/OD280 1.9-2.0), RNA was reverse transcribed into cDNA using the miScript II RT Kit (Qiagen, Germany). Obtained cDNA was stored at −20°C for further experiment. An ABI7300HT instrument (Applied Biosystems, USA) was applied to measure the level of the mRNAs by the SYBR Green PCR Kit (Qiagen, Germany). Each experiment was performed in triplicate. The primers of miR-451 and miR-506 were purchased from Sangon Inc. (Shanghai, China). *β*-Actin was applied to normalize mRNA expression, which was analyzed by the 2^−ΔΔCt^ method.

### 2.3. Statistical Analysis

SPSS 20.0 software (SPSS Inc., USA) and GraphPad Prism 8.0 software (GraphPad Software, Inc., USA) were adopted to analysis the date. The data are presented in the form of mean ± standard deviation. The *t*-test was performed to compare the difference between groups. The chi-square test was adopted to explore the relationship between miR-451 and miR-506 expression with clinical characteristics of breast cancer patients. The receiver operating characteristics (ROC) assay was conducted to measure diagnostic performance of miR-451 and miR-506 for breast cancer patients. The Kaplan–Meier method and log-rank test were used to conduct survival analysis for breast cancer patients with different miR-451 and miR-506 expression. *P* < 0.05 can be considered as the difference between groups is significant.

## 3. Results

### 3.1. miR-451 and miR-506 Were Downregulated in Breast Cancer Tissues

In order to explore serum miR-451 and miR-506 expression in breast cancer, qRT-PCR was conducted initially to detect their expression. We found that compared with the healthy samples, miR-451 and miR-506 expression was decreased in the serum of breast cancer patients (Figures 1(a) and 1(b)). Subsequently, the expression levels of miR-451 and miR-506 were examined in breast cancer tissues and paracancerous tissue. Consistent with the results in serum samples, miR-451 and miR-506 expression decreased in breast cancer tissues compared with paracancerous tissue (Figures 1(c) and 1(d)).

### 3.2. Relationship between miR-451 and miR-506 Expression with Clinical Characteristics of Breast Cancer Patients

According to the expression level of miR-451 or miR-506 in serum, breast cancer patients were divided into two groups (low miR-451 expression (*n* = 49) vs. high miR-451 expression (*n* = 39) groups; low miR-506 expression (*n* = 45) vs. high miR-506 expression (*n* = 43) groups). Subsequently, the association between miR-451 and miR-506 expression and clinical characteristics of breast cancer patients was explored by the chi-square test. Results showed that the miR-451 and miR-506 expression were both positively associated with lymph node metastasis and TNM stage (Table 1). There was no significant correlation between miR-451 or miR-506 expression and other clinical indexes, including age, tumor size, PR status, ER status, and human epidermal growth factor receptor 2 (HER-2) status.

### 3.3. Diagnostic Performance of miR-451 and miR-506 Expression for Breast Cancer Patients

The ROC analysis was conducted to further prove the accuracy of miR-451 and miR-506 in breast cancer diagnosis. The area under the curve (AUC) of the serum miR-451 and miR-506 was 0.850 and 0.832, respectively (Figures 2(a) and 2(b)), indicating miR-451 and miR-506 could be considered as a new serum prognostic biomarker of breast cancer.

### 3.4. Relationship between miR-451 and miR-506 Expression with Prognosis in Breast Cancer Patients

Additionally, the Kaplan–Meier method was applied to figure out the relationship between miR-451 and miR-506 expression and the five-year survival rate of breast cancer patients. The result showed that breast cancer patients with low miR-451 and miR-506 expression had higher five-year survival rate compared with those patients with miR-451 and miR-506 high expression (Figures 3(a) and 3(b)).

## 4. Discussion

Breast cancer is one of the most common causes of cancer deaths in the world, leading to 63,000 deaths in 2018, which causes great physical, psychological, and economic pressure to the majority of patients [19]. Patients with advanced breast cancer often suffer from dyspnea, bone pain, weight loss, ulcers, and other problems, leading to poor quality of life. Nowadays, there are many cancer treatment methods, such as radiotherapy, chemotherapy, endocrine therapy, and so on. However, the mortality of breast cancer is still high, and the quality of life of advanced patients is poor. Therefore, early diagnosis of breast cancer is extremely important. Although the overall survival rate of breast cancer patients has increased obviously, the quality of life of patients with advanced breast cancer is still very poor, suffering from bone pain, dyspnea, and ascites. In recent years, studies have confirmed that miRNA is involved in many biological activities, especially the cell proliferation and invasion of malignant tumors, and can be used as a therapeutic target for cancer treatment [20]. The important role of miRNA in the early diagnosis and prognosis of a series of cancers has been confirmed, such as miR-223 [21], miR-30a-5p [22], and miR-105 [23].

In this study, we evaluated the clinical diagnosis value and prognosis of miR-451 and miR-506 in breast cancer. We first detected the expression levels of miR-451 and miR-506 in the serum of breast cancer patients and healthy volunteers. The results showed that the expression of miR-451 and miR-506 in breast cancer patients was significantly lower than that in the control group. Consistent with the results in serum samples, miR-451 and miR-506 expression decreased in breast cancer tissues compared with paracancerous tissue. In addition, we found that miR-451 and miR-506 expression was both associated with lymph node metastasis status and TNM stage. These results imply that miR-451 and miR-506 may be a tumor suppressor gene and may be of great significance for clinical prognosis and diagnosis of breast cancer. Similar results have been confirmed in other cancers, such as nonsmall cell lung cancer [24], gastric cancer [25], colon cancer [26], and so on. In addition to the differential expression of miRNAs and its effect on cell proliferation and invasion in malignant tumors, they have also been widely confirmed to play an important role in clinical diagnosis and prognosis. For instance, serum exosomal miR-506 was considered as a potential diagnostic and prognostic biomarker of colorectal cancer [27]. Low expression of miR-145 tended to be positively correlated with lymphatic metastasis, clinical staging, and shorter overall survival of patients [28].

To further analyze the diagnostic accuracy of miR-451 and miR-506 as a marker of breast cancer, we conducted ROC analysis to compare breast cancer patients and healthy individual. The AUC of the serum miR-451 and miR-506 was 0.850 and 0.832, respectively, suggesting serum miR-451 and miR-506 as a new diagnostic method for breast cancer showing high diagnostic accuracy. This indicates that miR-451 and miR-506 may be a candidate diagnostic biomarker. Furthermore, survival analysis suggested that low miR-451 and miR-506 expression was relevant to favorable prognosis of breast cancer. Therefore, miR-451 and miR-506 were considered as an independent prognostic biomarker of breast cancer.

In conclusion, the level of miR-451 and miR-506 expression showed high diagnostic accuracy for distinguishing breast cancer patients and healthy people. miR-451 and miR-506 could be used as the biomarker for the diagnosis and prognosis of breast cancer.

## Figures and Tables

**Figure 1:** miR-451 and miR-506 expression was detected by qRT-PCR. (a)-(b) Serum miR-451 and miR-506 levels significantly lower in breast cancer patients than those in the control group. (c)-(d) miR-451 and miR-506 expression significantly lower in breast cancer tissues than those in the control group.

**Figure 2:** (a) Receiver operating characteristics (ROC) curve analysis of serum miR-451 in all breast cancer patients. (b) ROC curve analysis of serum miR-506 in all breast cancer patients.

**Figure 3:** Kaplan–Meier survival analysis of five-year survival rate according to serum miR-451 (a) and miR-506 (b) levels.

**Table 1:** Association of miR-451 and miR-506 with clinicopathological features of breast cancer patients.

Parameters	*N*	miR-451 expression				miR-506 expression			
		Low (*n* = 49)	High (*n* = 39)	*χ* ^2^	*P*	Low (*n* = 45)	High (*n* = 43)	*χ* ^2^	*P*
Age, years				0.947	0.330			1.366	0.243
≤40	32	20	12			19	13		
>40	56	29	27			25	31		
Tumor size, cm				1.741	0.187			1.092	0.296
≤3	36	18	18			16	20		
>3	52	31	21			29	23		
LNM				4.503	0.034			6.527	0.011
Negative	43	19	24			19	24		
Positive	45	30	15			28	17		
ER				3.215	0.073			1.31	0.252
Negative	34	23	11			20	14		
Positive	54	26	28			24	30		
PR				1.108	0.292			0.682	0.409
Negative	33	16	17			15	18		
Positive	55	33	22			30	25		
HER-2				0.485	0.486			0.158	0.691
Negative	51	30	21			29	22		
Positive	37	19	18			18	19		
TNM stage				4.946	0.026			4.632	0.031
I-II	47	21	26			19	28		
III-IV	41	28	13			25	16		

LNM, lymph node metastasis; ER, estrogen receptor; PR, progesterone receptor; HER-2, human epidermal growth factor receptor 2.

## Data Availability

The data used to support the findings of this study are available from the corresponding author upon request.
